# Effectiveness of Quantitative Shear Wave Elastography for the Prediction of Axillary Lymph Node Metastasis

**DOI:** 10.1155/2022/8769889

**Published:** 2022-06-28

**Authors:** Yingying Cheng, Guofu Li, Hui Jing, Shasha Yuan, Lei Zhang, Wen Cheng

**Affiliations:** ^1^Department of Ultrasound, Harbin Medical University Cancer Hospital, Harbin, China; ^2^Department of Neurosurgery, Harbin Medical University Cancer Hospital, Harbin, China

## Abstract

**Objective:**

Invasive breast cancer can be metastasized through axillary lymph nodes (LNs). This study was to evaluate the effectiveness of quantitative shear wave elastography (SWE) to predict axillary LN metastasis, which also provides prognostic implication of SWE as a histopathologic element of invasive breast cancer.

**Methods:**

72 prospectively enrolled patients received B-mode ultrasound (BUS) and SWE, and the elasticity index (EI) of SWE at the stiffest part of lymph nodes (LNs) was measured. EI of SWE was closely associated with pathologic results and the histopathologic elements. The receiver operating characteristics (ROC) curve was drawn to evaluate the optimal cut-off value for the assessment of disease severity.

**Results:**

A significantly longer short-axis diameter and a larger maximal cortex were observed in malignant LNs than that in healthy LNs. The absence of the hilum was associated with metastatic LNs. The EI of SWE varied markedly between the benign and malignant LNs. The combination of *E*_max and_ BUS showed higher area under the curve (AUC) than BUS alone to predict metastatic LNs (0.7762 vs. 0.7230). EI of SWE in malignant lymph nodes those with extranodal extension are higher than those without extranodal extension.

**Conclusions:**

Quantitative SWE provides a viable alternative for the assessment of axillary LN and shows great potential to predict pathological prognostic elements of metastatic axillary LNs in invasive breast cancer. Joint use of SWE and BUS allows examination of the predictive outcome of BUS for axillary lymph node metastasis in invasive breast cancer.

## 1. Introduction

The correlation between axillary lymph node metastasis and prognostic of invasive breast cancer remains elusive. Lymph node (LNs) metastasis affects prognosis and treatment decisions [1, 2], so assessment of lymph node metastasis in breast cancer is of great importance. Clinical results revealed that axillary lymph node metastasis showed low sensitivity of 45.4% to 68% [3–5]. Axillary ultrasonography is an important tool for lymph node metastases inspection. However, the sensitivity of axillary ultrasonography only ranges from 35% to 82%, with specificity being 73% to 97.9% [6–9]. The average sensitivity of ultrasound-guided core needle biopsy (CNB) is 89.8% for suspicious axillary lymph nodes, 60.3% for large metastases, and 26.7% for micrometastases [10]. It is obvious that the current detection of lymph node metastasis may still result in missed diagnosis. Compared with axillary lymph node dissection (ALND), sentinel lymph node biopsy (SLNB) features higher precision and less invasiveness as a treatment. However, SLNB may give rise to complications such as lymphedema and seroma formation [11]. Therefore, there exists a need to explore a noninvasive imagological examination to predict metastatic axillary lymph nodes of invasive breast cancer.

The stiffness of LNs can be objectively assessed by ultrasound elastography given the different stiffness between benign and malignant LNs [12, 13]. Nonetheless, the results of strain elastography are impacted by the proficiency of the radiologists and the variations of measured organizational elasticity [14–17]. With the advancement in medical technology, shear wave elastography (SWE) was developed to overcome the relevant limitations by providing quantitative statistics about tissue elasticity. SWE is a quantitative elastography technique that generates sheer wave using professional sensors and ultrafast ultrasonic tracking technology to obtain the velocity of induced shear wave and the real-time output displayed on tissue stiffness based on elastic diagram [18–21]. Recent studies reported the application of SWE for inspection of many organs such as the breast, thyroid, prostate, cervix, and liver [19,22–24]. SWE is scarcely used to predict axillary lymph node metastasis in invasive breast cancer. This study was undertaken to assess the effectiveness of quantitative SWE to predict axillary LNs metastasis in invasive breast cancer and to predict the correlation of elasticity index (EI) of SWE with histopathologic elements of axillary lymph node metastasis.

## 2. Materials and Methods

This retrospective study was approved by the ethics committee of the Cancer Hospital of Harbin Medical University, Harbin, China. Undersigned informed consent was obtained from all patients.

### 2.1. Patients

Women with ultrasound-detected abnormalities and those with symptoms were included in the study [25]. Axillary lymph nodes were determined as abnormal (round, absence of fat hilus, calcification, cystic changes, cortical heterogeneity, and confusion of vascular pattern) [26], whereas they were deemed benign without the above-mentioned. From January 2014 to February 2015, 72 patients (115 lymph nodes) with invasive breast cancer underwent routine B-mode ultrasonography (BUS) and SWE examination before operation.

The enrolled patient underwent conventional BUS and SWE of the enlarged or suspicious axillary lymph nodes, and the imaging was performed with the patients in the supine or slightly (30°) left lateral decubitus position with the right arm elevated above the head. BUS and SWE were performed using the ultrasound imaging equipment produced by AIKE in Provence, France, with a 15-4 MHz linear array transducer SWE and gray-scale ultrasound images were obtained, using the default elasticity settings for penetration, persistence, smoothing, and kilopascal (kPa) display scale (0–180 kPa). On SWE, a square frame was used to include axillary lymph nodes and surrounding tissue cells. LNs with a depth over 3 cm were excluded given the signal loss in SWE at such depth. Red and blue areas on SWE correspond to stiff and soft regions, respectively. Three or more SWE/US cineloop fragments were obtained by using different parts of each node. The duration of the obtained fragments was displayed for 10 seconds, and the sensor remained still during capture. For each cineloop, the first few seconds were omitted as the elastogram during which is not stable, and single still images, with the least artifacts, such as vertical linear color bands passing through different tissues or other high hardness color parts in the surrounding fascia, were selected. For each selected still image, the hardest part of lymph node cortex and portal was selected by visual inspection, on which a circular electronic region of interest or Q-box was placed [27]. The software determines the relevant index for each Q-box, in which the maximum (*E*_max_) and average (emean) and minimum (*E*_min_) elastic values (kPa) were analyzed (Figure 1). The elastic index (EI) of surrounding muscles was calculated to clarify the Emean comparison value (Emean-m) of LNs and surrounding muscles. By moving a delineated region of interest (ROI) over the color map, the values of elasticity were obtained. ROI were placed of stiffest areas on color maps to obtain max ROI, mean ROI, min ROI, and mean-m ROI for analysis [28]. The selection of the highest value to measure the entire lymph node determines the absence of complete infiltration of the lymph node by tumor cells or spatial heterogeneity due to tumor necrosis.

### 2.2. Histopathologic Diagnosis

Of 61 suspicious axillary lymph nodes, 43 were treated with surgery and 18 with neoadjuvant chemotherapy after CNB. Of the remaining 54 LNs, 38 were treated with surgery or SLNB due to discordant ultrasound results or clinician request, and 12 LNs had ultrasound follow-up for 6 to 9 months. To facilitate accurate comparison between imaging results and histopathological results, the tissues were fixed by 10% formalin, paraffin embedded and sectioned, followed by eosin and hematoxylin staining. The histopathological diagnosis of LNs was reviewed, which was closely related to SWE results. The histopathological manifestations of metastatic LN were determined by the ratio of surgical specimens and the number of metastatic LN divided by the number of anatomical LN (metastatic ln/anatomical LN).

### 2.3. Statistical Analysis

Data analyses were performed based on the histopathologic results from LN dissections. SWE elasticity indices (*E*_max_, E_mean_, *E*_min_, and E_mean-m_) were closely associated with the pathological and histopathological results of metastatic lymph nodes, which was obtained with Student's *t*-test age's differences and short-axis diameter between benign and metastatic LNs. Wilcoxon rank sum test was used to determine the long/short-axis ratio, maximal cortex, *E*_max_, Emean and Emin between benign and metastatic LNs. The *t*-test was used to determine the differences in Emean-m between benign and metastatic LNs. Chi-square experiment was applied to clarify the different selection methods for the absence and presence of hilum between benign and metastatic LNs. Spearman correlation coefficient and Student's *t*-test were used to analyze the correlation between EI of SWE and histopathological results of metastatic LNs [29]. The ability of EI of SWE and BUS category values to differentiate between benign and malignant LNs was evaluated using the ROC curve. After obtaining the best cut-off data, x2 test was used to measure the sensitivity, specificity, accuracy, positive predictive value (PPV), and negative predictive value (NPV). The generalized estimation equation was adopted to effectively analyze the optimal cut-off data based on the logistic regression model, and assessments were performed on the basis of the comparative analysis of the area under the curve (AUC) value and 95% confidence interval (CI) diagnostic performance of ultrasonic classification. The statistical analysis was implemented in SAS version 9.2 (Cary SAS Institute, North Carolina, USA). *P* < 0.05 was set as the cut-off for statistical significance.

## 3. Results

### 3.1. Correlation of SWE and Pathologic Results of LNs

115 LNs in 72 patients were examined by BUS and SWE from January 2014 to February 2015.115 LNs were dissected by ultrasound-guided labeling. 70 cases (60.9%) were metastatic lymph nodes, and 45 cases (39.1%) were benign lymph nodes. Malignant LNs were associated with a longer short-axis diameter and a larger maximal cortex versus healthy LNs (Table 1; *P* < 0.0001). The absence of the hilum was associated with metastatic LNs (Table 1; *P* < 0.0001). *E*_max_, *E*_mean_, *E*_min,_ and Emean-m were significantly larger in malignant LNs than in healthy LNs (Table 1; *P* < 0.0001).

The diagnostic performances of *E*_max_, *E*_mean_, *E*_min,_ and *E*_mean-m_ using sensitivity, specificity, accuracy, PPV, NPV, and estimated critical value were used to predict the actual situation of metastasis and distinguish benign lymph nodes from metastatic lymph nodes 21.10 kPa (*E*_max_), 13.10 kPa (*E*_mean_), 9.00 kPa (*E*_min_), and 1.58 (E_mean-m_), as presented in Table 2. The comparison of AUC values between SWE and BUS is shown in Table 3. AUC values of *E*_max_, *E*_mean_, *E*_min,_ and *E*_mean-m_ were not different from those of BUS (*P* > 0.05). However, AUC of *E*_max_ plus BUS is higher than that of BUS alone (*P*=0.0208; Table 3).

### 3.2. Correlation between EI of SWE and Histopathology of Metastatic LNs

Table 4 presents the relationship between EI of SWE and histopathological results of metastatic LN, in which there is a relationship between EI of SWE of *E*_max_, *E*_mean_, *E*_min,_ and *E*_mean-m_ and the number of metastatic LNs, and the ratio of malignant LNs/dissected LNs and the L/S (Long-/short-axis ratio) were not significantly different (*P* < 0.05). EI of SWE in malignant lymph nodes those with extranodal extension are higher than those without extranodal extension (*P* < 0.0001 for *E*_max_, *E*_mean,_ and *E*_min_; Table 4).

## 4. Discussion

Lymph node metastasis compromises the outcome of surgical treatment, radiotherapy, and neoadjuvant therapy, so the prediction of axillary lymph node status is of great significance in the prognosis of patients with invasive breast cancer. The 5-year survival of patients with positive lymph nodes is 40%, which is lower than that of patients without lymph node metastasis [30]. Previous studies have reported that BUS features including low long-to-short-axis diameter ratio, heterogeneous cortical thickening, and absence of fat gates and peripheral blood flow are associated with lymph node metastasis. Several studies have investigated the significance of quantitative SWE in patients with breast cancer [31, 32]. However, SWE has not been evaluated for metastatic LN in invasive breast cancer.

Here, metastatic LNs were associated with a longer short-axis diameter and a larger maximal cortex versus benign LNs, and the absence of hilum was associated with metastatic LNs. These results were similar to those from previous studies [33]. The present study found that EI of SWE of *E*_max_, *E*_mean_, *E*_min,_ and E_mean-m_ were significantly higher in malignant LNs when compared with benign LNs. In addition, the results showed the highest sensitivity (81.43%), accuracy (81.74%), and NPV (74%) with *E*_mean-m_ (cutoff lever of 1.58), highest specificity (93.33%), and PPV (94.23%) with *E*_max_ (cutoff lever of 21.10 kPa). These results are similar to the results of previous research [34]. The difference of diagnostic performance between BUS and SWE did not come up to the statistical standard. However, our study found *E*_max_ plus BUS outperformed BUS only (AUC 0.7762 vs. 0.7230; *P*=0.0208). These findings suggest that SWE may serve as an important auxiliary diagnostic tool for invasive breast cancer.

In this study, quantitative SWE may be closely related to histopathological prognostic factors of metastatic lymph nodes, and the ratio (L/S), number of malignant LNs, and the ratio of metastatic LN/dissected LN were not significantly correlated with the quantitative EI of SWE. However, the mean values of Emax, Emean, Emin, and Emean-m with extranodal infiltration and metastasis were significantly different from those without lymph nodes (44.35 ± 6.06 vs. 24.01 ± 8.46 kPa, 28.42 ± 8.81 vs. 25.71 ± 6.21 kPa, 16.59 ± 5.41 vs. 10.01 ± 3.61 kPa, and 2.71 ± 0.67 vs. 1.70 ± 0.41 kPa, respectively; *P* < 0.0001). These results were similar to those of previous studies and suggested that EI of SWE is available to help determine the degree of the benignity of LN to decide the use of surgery or neoadjuvant therapy for invasive breast cancer patients.

Real-time shear wave elastography, as a new concept for tissue hardness evaluation, overcomes the objective impacts such as the size and frequency of probe pressure in static/quasistatic elastography and features the advantages of good repeatability, rapidity, and no dependence.

There were several limitations in the current study. First, the number of our samples is small, and the follow-up duration was short. Furthermore, evaluation of factors affecting the elasticity measurements including degree, depth, size, and location of calcification in a single lymph node was absent. Second, SWE was performed in preoperative staging ultrasound in patients with invasive breast cancer, which may result in a selection bias. Third, the accuracy of the examinations used in this study was correlated with LNs removed in the surgery. However, the removed LNs herein were fixed in formalin which may lead to alterations in the sizes of the LNs. Finally, this study did not obtain a detailed correlation between the EI of SWE and histopathological elements of metastatic breast cancer in metastatic LNs. Future multicenter studies will be carried out with a larger sample size, a longer follow-up duration, and improvement of the above limitations to provide more convincing data.

## 5. Conclusions

Quantitative SWE provides a viable alternative for the assessment of axillary LN and shows great potential to predict pathological prognostic elements of metastatic axillary LNs in invasive breast cancer. Joint use of SWE and BUS allows examination of the predictive outcome of BUS for axillary lymph node metastasis in invasive breast cancer.

## Figures and Tables

**Figure 1:** Shear wave elastography (SWE) and B-mode ultrasonography (BUS) images of a metastatic axillary lymph node from an invasive breast cancer in a 56-year-old women. Findings consistent with malignancy on BUS included loss of hilar fat and cortical heterogeneous echogenicity (lower image). SWE was performed for the lymph node and a Q-box is placed over the stiffest region, as assessed by visual inspection. A 2-mm-size circular region of interest was selected at the stiffest portion and elasticity scores of 42.5 kPa (*E*_max_), 53.9 kPa (*E*_mean_), 23.8 kPa (*E*_min_), and 3.63 (*E*_mean-m_)were obtained. *E*_max,_ maximal elasticity score of the lesion; *E*_mean,_ mean elasticity score of the lesion; *E*_min,_ minimal elasticity score of the lesion; *E*_mean-m,_ ratio of *E*_mean_ mean of the lesions divided by *E*_mean_ of surrounding muscles.

**Table 1:** Statistic analysis between benign and malignant lymph nodes (*n* = 115).

Variable	Benign (*n* = 45)	Malignant (*n* = 70)	Statistic value	*P* value
Age (year)	53.31 ± 9.84	51.8 ± 9.04	0.84	0.4000^a^
Short-axis diameter (mm)	5.30 ± 1.50	11.5 ± 6.20	7.95	<0.0001^a^
Long/short-axis ratio	1.76(1.55,2.21)	1.585(1.34,2.08)	3.71	0.0541^b^
Maximal cortex (mm)	2.20(1.40,3.20)	5.20(2.30,7.20)	20.19	<0.0001^b^
Hilum			19.35	<0.0001^d^
Absent, *n* (%)	2.00 (4.4%)	31.00 (44.3%)		
Present, *n* (%)	43.00 (95.6%)	39.00 (55.7%)		
*E*_max_ (kPa)	16.80 (14.50,19.40)	25.45 (19.0,41.50)	46.12	<0.0001^b^
*E*_mean_ (kPa)	11.70 (9.90,12.60)	15.45 (13.20,24.70)	34.61	<0.0001^b^
*E*_min_ (kPa)	7.90 (6.50,9.80)	11.15 (9.00,13.80)	24.32	<0.0001^b^
*E*_mean-m_ (kPa)	1.36 ± 0.28	2.03 ± 0.61	−8.05	<0.0001^c^

*E*_max,_ maximal elasticity score of the lesion; *E*_mean,_ mean elasticity score of the lesion; *E*_min,_ minimal elasticity score of the lesion; *E*_mean-m,_ ratio of *E*_mean_ mean of the lesions divided by *E*_mean_ of surrounding muscles.^a^Student's *t* test.^b^Wilcoxon rank sum test.^c^Student's *t*' test.^d^Chi-square test.

**Table 2:** Diagnostic performance of BUS and SWE for predicting axillary lymph node metastasis.

Variables	Cutoff values	Sensitivity (%)	Specificity (%)	PPV (%)	NPV (%)	Accuracy (%)
BUS		75.71	68.89	79.10	64.58	73.04
*E*_max_	21.10	70.00	93.33	94.23	66.67	79.13
*E*_mean_	13.10	78.57	80.00	85.94	70.59	79.13
*E*_min_	9.00	75.71	68.89	79.10	64.58	73.04
*E*_mean-m_	1.58	81.43	82.22	87.69	74.00	81.74
BUS + *E*_max_	21.10	88.57	66.67	80.52	78.95	80.00
BUS + E_mean_	13.10	91.43	57.78	77.11	81.25	78.26
BUS + *E*_min_	9.00	91.43	51.11	74.42	79.31	75.65
BUS + E_mean-m_	1.58	95.71	60.00	78.82	90.00	81.74

BUS, B-mode ultrasound category; SWE, shear wave elastography; PPV, positive predictive value; NPV, negative predictive value; *E*_max,_ maximal elasticity score of the lesion;, *E*_mean,_ mean elasticity score of the lesion; *E*_min,_ minimal elasticity score of the lesion; *E*_mean-m,_ ratio of *E*_mean_ mean of the lesions divided by *E*_mean_ of surrounding muscles; BUS + *E*_max,_ combined use of *E*_max_ and BUS; BUS + *E*_mean_, combined use of *E*_mean_ and BUS; BUS + *E*_min,_ combined use of *E*_min_ and BUS; BUS + *E*_mean-m,_ combined use of *E*_mean-m_ and BUS.

**Table 3:** Comparison of diagnostic performances of BUS and SWE.

Parameters	AUC (95% CI)	*P* value (compared with BUS)
BUS	0.7230 (0.6379,0.8081)	
*E*_max_	0.8167 (0.7512,0.8821)	0.0574
*E*_mean_	0.7929 (0.7165,0.8692)	0.1913
*E*_min_	0.7230 (0.6379,0.8081)	1.0000
*E*_mean-m_	0.8183 (0.7455,0.8910)	0.0768
BUS + *E*_max_	0.7762 (0.6971,0.8553)	0.0208
BUS + E_mean_	0.7460 (0.6659,0.8261)	0.4756
BUS + *E*_min_	0.7127 (0.6318,0.7936)	0.7756
BUS + *E*_mean-m_	0.7786 (0.7024,0.8548)	0.0849

BUS, B-mode ultrasound category; SWE, shear wave elastography; AUC, area under the curve; CI, confidence interval; *P* value is for parameter compared with the ultrasound category; *E*_max,_ maximal elasticity score of the lesion; *E*_mean,_ mean elasticity score of the lesion; *E*_min,_ minimal elasticity score of the lesion; E_mean-m,_ ratio of E_mean_ mean of the lesions divided by E_mean_ of surrounding muscles; BUS + *E*_max,_ combined use of *E*_max_ and BUS; BUS + E_mean,_ combined use of E_mean_ and BUS; BUS + *E*_min,_ combined use of *E*_min_ and BUS; BUS + E_mean-m,_ combined use of E_mean-m_ and BUS.

**Table 4:** Correlation of Emean-m and histopathologic factors in metastatic LN of invasive breast cancer.

Variables	No. of metastatic LN^#^		Ratio of metastatic LN/dissected LN^#^		L/S^#^		Extranodal extension^*∗*^		
	Coefficient	*P* value	Coefficient	*P* value	Coefficient	*P* value	Without extension	With extension	*P* value
*E*_max_	0.0657	0.6573	0.0662	0.6550	−0.1238	0.1876	24.01 ± 8.46	44.35 ± 6.06	<0.0001
*E*_mean_	0.2037	0.1650	0.1350	0.3602	−0.0392	0.6772	15.71 ± 6.21	28.42 ± 8.81	<0.0001
*E*_min_	0.0970	0.5120	0.2136	0.1449	0.0237	0.8018	10.01 ± 3.61	16.59 ± 5.41	<0.0001
*E*_mean-m_	0.1574	0.2852	0.1159	0.4328	−0.0082	0.9309	1.70 ± 0.41	2.71 ± 0.67	<0.0001

SWE, shear wave elastography; EI, elasticity indices; LN, lymph node; *E*_max,_ maximal elasticity score of the lesion; *E*_mean,_ mean elasticity score of the lesion; *E*_mi,_ minimal elasticity score of the lesion; *E*_mean-m,_ ratio of *E*_mean_ mean of the lesions divided by *E*_mean_ of surrounding muscles. ^#^Spearman correlation coefficient. ^*∗*^Student's *t* test.

## Data Availability

The data sets used and analyzed in this study can be obtained from the corresponding authors in combination with specific requirements.
